# Role of Posttreatment Nursing Based on Functional Magnetic Resonance Imaging in Breast Cancer Patients with Lymphedema

This article has been retracted.

**DOI:** 10.1155/2022/5224288

**Published:** 2022-09-06

**Authors:** Ru Sun, Haihong Li, Xin Wang, Jun Shen, Lingzhi Guo, Wenwen Sun

**Affiliations:** ^1^Department of Breast Surgery, The First People's Hospital of Lianyungang, Lianyungang 222002, Jiangsu Province, China; ^2^Department of Nursing, The First People's Hospital of Lianyungang, Lianyungang 222002, Jiangsu Province, China; ^3^Department of Otorhinolaryngology Head and Neck Surgery, The First People's Hospital of Lianyungang, Lianyungang 222002, Jiangsu Province, China

## Abstract

Breast cancer is the tumor disease with the highest incidence in women, especially lymphedema after treatment, which seriously affects the quality of life of women. In order to improve the nursing quality of breast cancer patients, medical staff uses functional magnetic resonance imaging (fMRI) to intervene in breast cancer patients, which greatly improves the recovery speed of patients. In this paper, functional magnetic resonance imaging based on the image registration method is proposed and applied to the follow-up of patients with breast cancer lymphedema after treatment. The powerful imaging effect allows doctors to timely and accurately judge the condition of the patient's lesions after treatment, which is conducive to nursing care. The experimental results of this paper show that the total number of serious patients in group *A* before the experiment is 25, accounting for 83.3%. After the experiment, the total number of severe cases was 24, accounting for 80%, indicating that the nursing measures of group *A* did not have a great effect. The total number of severe cases in group *B* before the experiment was 27, accounting for 90%. The total number of severe cases after the experiment was 10, accounting for 33.3%. The effect after the experiment was significantly higher than that before the experiment, indicating that the nursing program of group *B* played a great role.

## 1. Introduction

Clinical epidemiology shows that the incidence of breast cancer in China is about 170,000 each year, ranking second among female malignant tumors, and the number of deaths is also increasing year by year. In recent years, patients not only pay attention to the survival period but also pay more and more attention to the quality of life. For patients with lymphedema after breast cancer surgery, the degree of lymphedema is proportional to the degree of its harm. Lymphedema is a common complication after axillary dissection characterized by regional enlargement of one arm. After the occurrence of lymphedema, the quality of life of patients is seriously affected due to limited range of motion of the arm, pain, abnormal appearance, heaviness and tightness of the upper arm, repeated infections, and induction of lymphosarcoma of the upper extremity. Under the premise of ensuring the treatment effect and improving the survival period, it has become a new research direction and focuses on ensuring the postoperative quality of life of patients as much as possible. Most studies have shown that the 10-year survival rate of patients with early breast cancer after correct nursing is more than 90%, and there is no significant difference in the long-term survival rate after fMRI treatment and modified radical mastectomy.

People's attention to health and the progress of treatment technology make breast cancer detected earlier and better treated. As a result, the survival time of patients has been gradually prolonged, and the 5-year survival rate of breast cancer in China has increased to 73%. Therefore, more and more researchers began to pay attention to the quality of life of breast cancer patients after surgery. Breast cancer lymphedema has also begun to receive attention as a major factor affecting the quality of life of patients after breast cancer surgery. In recent years, functional magnetic resonance imaging (fMRI) technology developed based on MRI technology has become an important auxiliary method for breast cancer diagnosis. In breast cancer, enhanced breast CT and breast fMRI are commonly used auxiliary methods for the diagnosis of breast cancer in clinical practice. Clinical studies have shown that compared with the use of enhanced CT imaging, the use of fMRI examination has higher diagnostic accuracy, and fMRI imaging examination has the advantages of no radioactive radiation and high resolution, and it can also obtain anatomical image information of breast lymph nodes. The innovation of this paper is to apply fMRI to patients with breast cancer-related lymphedema after surgery to explore the effect of fMRI on swelling of the affected limb, lymphedema-related symptoms and distress, and on the quality of life.

## 2. Related Work

With the increasing incidence of breast cancer in recent years, people have paid more and more attention to its treatment and postoperative care. Ziv et al. found family history to be a known risk factor for breast cancer. Two genes associated with significantly increased breast cancer risk have been identified, but mutations in these genes are relatively rare, and a recent study suggests that the cause of reduced biological activity may be associated with increased cancer risk [1]. Lautrup et al. described prognostic parameters in male breast cancer patients. Survival and mortality compared with female breast cancer patients over the same period were also analyzed. The data comes from the DBCG database. He found significant differences in survival and mortality between the two sexes [2]. Retsky et al. found that surgical removal of primary breast cancer accelerates recurrence in some premenopausal patients with positive lymph nodes. For untreated patients, these accelerated recurrences occurred within 10 months of surgery. The mechanism he proposed is to stimulate angiogenesis in dormant micrometastases [3]. Yuka et al. found that the prognosis of breast cancer is poor due to frequent recurrence of breast cancer. The Androgen receptor (AR) is involved in the pathogenesis of breast cancer, but its role is still unclear. His aim was to investigate the expression of AR and its relationship to the clinicopathological features of breast cancer [4]. Harris and Small discovered that intraoperative radiotherapy (IORT) for early breast cancer is a technique used for partial breast irradiation. There are several clinical techniques available for performing breast IORT. IORT usually refers to the delivery of a single dose of radiation around the tumor bed within the immediate intraoperative time frame and the safety and efficacy of breast IORT in patients with early breast cancer [5]. Scholars have realized that breast cancer is a kind of cancer with a high incidence among women, which greatly reduces women's quality of life and threatens their lives. Scholars have also found that breast cancer has a high probability of recurrence after surgery, but they have not proposed how to reduce the recurrence rate.

The fMRI technology developed on the basis of magnetic resonance imaging has received extensive attention and research due to its noninvasive and precise ability to locate lesions. Alexis et al. used functional magnetic resonance imaging (fMRI) to examine the neural basis of language control. Brain responses generated during simultaneous interpretation (SI) were compared with those generated during simultaneous repetition [6]. Liu et al. found that global signals can be used to cancel global changes in functional magnetic resonance imaging (fMRI). However, there is considerable controversy over its use due to potential biases that may be introduced when studying fMRI [7]. Ali et al. found that a multivariate Granger causal analysis could be performed with resting-state functional magnetic resonance imaging (rs-fMRI) data to calculate various directed graph measures. It was used as the original feature set for machine learning algorithms, and the classification accuracy reached 93.3% [8]. Chen et al. found that in the field of resting-state functional magnetic resonance imaging (R-fMRI), concerns have been raised about the reproducibility of findings. He comprehensively assessed the reproducibility of widely used R-fMRI metrics and systematically investigated the impact of small sample sizes [9]. In view of the high recurrence rate of breast cancer, scholars have proposed fMRI technology, which can accurately identify the lesions, locate the lesions, and can affect the postoperative care of patients with breast cancer lymphedema. But scholars do not have specific experiments to prove that this method can effectively carry out nursing.

## 3. Functional Magnetic Resonance Imaging Technology Based on Image Registration

### 3.1. Basic Algorithm Based on Image Registration Method

Breast cancer is one of the most important tissues and organs in the human body, and breast cancer is currently two of the most common malignant tumors in clinical practice and it occupies a high place among various types of tumor death causes [10]. Early treatment and care of breast cancer patients is the key to prolonging their survival time, so nursing care after breast cancer lymphedema treatment has attracted more and more attention. Traditional care for lymphedema in breast cancer is shown in Figure 1.

As shown in Figure 1: Postoperative lymphedema in breast cancer patients has a comprehensive impact on the body, which will reduce the patient's immunity and increase the possibility of infection. If lymphedema occurs and is not managed and treated over time, it will gradually worsen and become irreversible. If moderate or severe lymphedema develops, patients should undergo surgery when conservative treatment fails. The most commonly used surgical methods are liposuction and lymphatic-vein anastomosis. Surgery can reduce the volume of the affected limb and symptoms related to lymphedema, but surgery cannot completely cure lymphedema, and there will be swelling and the risk of reswelling after surgery [11]. Therefore, methods to promote lymph flow, avoid increased lymph production after surgery, promote postoperative rehabilitation of affected limbs, maintain postoperative outcomes, reduce symptoms associated with lymphedema, and take effective countermeasures to improve patients' quality of life are particularly important. Functional magnetic resonance imaging is an emerging neuroimaging modality that uses magnetic resonance imaging to measure hemodynamic changes caused by neuronal activity. The advantages of fMRI technology are shown in Figure 2.

As shown in Figure 2, the urgent need in the medical field further promotes the development of fMRI technology, and some pathological applications have begun to emerge, such as the use of diffusion imaging and perfusion imaging to diagnose cerebral ischemia. With the development of fMRI technology, it is widely used in breast cancer detection. Usually, the resolution of gland tissue in imaging examination is not enough, and dynamic contrast-enhanced fMRI imaging has a good imaging effect, which is especially helpful in determining whether small breast cancer is associated with breast hyperplasia. At the same time, dynamically enhanced fMRI has a good imaging effect on the deep breast masses that are difficult to distinguish from other images, so it can greatly reduce the missed diagnosis rate and misdiagnosis rate. Dynamic contrast-enhanced fMRI imaging is also dynamic and can well image the blood perfusion in the lesion [12].

Image registration is the process of matching and superimposing two or more images acquired at different times, different sensors, or under different conditions. Image registration is an important image processing technology that has important applications in many fields, such as computer vision and medical images. However, during the imaging process, the anatomical position between the images of the same slice at different times is biased due to the patient's voluntary movement and the displacement and deformation of the breast. This brings difficulties to the subsequent work such as benign and malignant discrimination, so it is imperative to register images. The image registration is shown in Figure 3.

As shown in Figure 3, whether it is feature-based or grayscale-based, image registration must establish a corresponding transformation model, especially for 3D images. In the transformation process, the transformation formula of the point $\left[\begin{array}{c} a_{1}\\ b_{1} \end{array}\right]$through the rigid body transformation to the point $\left[\begin{array}{c} t_{a}\\ t_{b} \end{array}\right]$is the following formula:

(1) $$\begin{array}{c} \left[\begin{array}{c} a_{1}\\ b_{1} \end{array}\right]=\left[\begin{array}{cc} \cos\;\theta & \pm \;\sin\;\theta \\ \mp \sin\;\theta & \cos\;\theta \end{array}\right]\left[\begin{array}{c} x\\ y \end{array}\right]+\left[\begin{array}{c} t_{a}\\ t_{b} \end{array}\right]\text{.} \end{array}$$

Among them, *θ* is the rotation angle and $\left[\begin{array}{c} t_{a}\\ t_{b} \end{array}\right]$ is the translation vector.

Due to the complexity of the deformation of human tissues and organs in medical images, nonrigid registration transformation is often used for medical image registration, and the commonly used spatial transformations include linear transformation and nonlinear transformation. Nonrigid registration based on free deformation is a traditional and popular nonrigid registration method. Among them, the more commonly used nonlinear transformations include the transformation model based on the thin plate spline function and the transformation model based on the *B*-spline function [13].

SPM, or Statistical Parametric Plot, is also the final output of this software. SPM is a method of statistical parameters, and it is also the result of the final processing and analysis of the software package. Its statistics are very powerful. SPM mainly processes and analyzes fMRI images and obtains statistically significant conclusions by comparing different image results between subjects or within subjects [14]. The overall schematic diagram of SPM processing fMRI data is shown in Figure 4.

As shown in Figure 4, specifically, a specific experimental design is used to make the subjects try to accept a certain stimulus or perform a certain task. Then, a series of processing and statistical analysis is performed on the acquired fMRI data to obtain the brain function activation area of the stimulus of interest [15, 16].

Thin-plate spline function is an interpolation algorithm that is used for image deformation, etc. and can drive the image to change through a small number of control points. The transformation of the thin plate spline function can be represented by the linear combination of affine transformation and radial basis function, and the transformation function is as follows:

(2) $$\begin{array}{c} f\left(A\right)=AX+B+\overset{n}{\underset{I=1}{\sum }}W_{I}I\left(\left|P_{I}-A\right|\right)\text{.} \end{array}$$

Among them, *X* is a coordinate vector, *A* and *B* define an affine transformation, *I* is a radial basis function, and there is formula (3) for a two-dimensional image:

(3) $$\begin{array}{c} U\left(r\right)=r^{2}\;\log\;r^{2}\text{.} \end{array}$$

According to the definition based on *B*-spline, the expression of the deformation *T* of the two-dimensional image in the two-dimensional space can be obtained, and the two-dimensional space can be expressed as follows:

(4) $$\begin{array}{c} \Omega =\left\{\left(a,b\right)\left|0\leq a≺A,0\leq b≺B\right.\right\}. \end{array}$$

Represents a grid space composed of control points *b* with a spacing of *a*. By moving the grid control points, the space of the surrounding neighborhood can be deformed by nonrigid displacement [17]. At the same time, because the *B*-spline has good local control ability when a control point of the grid changes, it will only cause the change of several surfaces adjacent to the point and will not affect the entire image [18].

FFD transformation based on *B*-spline belongs to a grid-type nonrigid deformation model. It uses the position of grid points to calculate the coordinate offset of each pixel point and finally resamples the pixels of the image according to the coordinate offset to realize its nonrigid deformation. The nonrigid registration algorithm based on the *B*-spline FFD model is applied to the registration of medical images. In order to solve the problem of the distortion of the lesion area during registration, some scholars use the FFD model based on the *B*-spline curve to describe the local deformation of breast dynamic enhanced MRI, as shown in the following formula:

(5) $$\begin{array}{c} E_{smooth}=\frac{1}{V}{\left(\frac{\partial^{2}T}{\partial a^{2}}\right)}^{2}\text{.} \end{array}$$

Among them, *V* represents the volume of the 3D image, and *T* represents the deformation field. The mutual information registration is realized, and the image registration measurement curve and the registered image are obtained by normalizing the mutual information registration. The normalized mutual information is used as the similarity measure in the registration, and the similarity in the registration is shown in the following formula:

(6) $$\begin{array}{c} E_{similarity}=\frac{H\left(A\right)+H\left(B\right)}{H\left(A,B\right)}\text{.} \end{array}$$

The final registration objective function is shown in the following formula:

(7) $$\begin{array}{c} E=-E_{similarity}+kE_{smooth}\text{.} \end{array}$$

Among them, *k* is the weight parameter. By minimizing the registration objective function, the optimal deformation field can be solved. However, when the mutual information is maximized in the solution process, the lesion area is inevitably distorted due to the grayscale variation between the images [19]. The registration objective function is actually to find a set of optimal parameters of the objective function, which involves finding the minimum or maximum value of the objective function.

The bending energy function based on *B*-spline FFD is used as a regular term to register medical images, and the obtained registration objective function is shown in formula (8), and the gradient descent method is used to solve the objective function [20]. Gradient descent is simply a method of finding the minimization of the objective function.

(8) $$\begin{array}{c} E=\min\;\left[\frac{1}{2}\sum \log\;\left(\frac{d^{2}}{\delta }+1\right)+\frac{k}{s}{\left(\frac{\partial^{2}T}{\partial a^{2}}\right)}^{2}\right]\text{.} \end{array}$$

In the formula, *T* represents the area of the two-dimensional image. The registration algorithm is robust to grayscale changes and can well model the deformation of the lesion area in medical images.

### 3.2. Removal of Offset Fields in Medical Images

The offset field is caused by the inconsistency of the grayscale of the MRI image due to the inhomogeneous magnetic field. The existence of the offset field greatly affects the accurate segmentation and subsequent processing of tissues and organs. Before further analysis and processing of medical images, image preprocessing is required to remove the offset field. The existence of the offset field in medical images not only brings trouble for doctors to diagnose diseases but also brings difficulties to computer automatic image processing technology. It has a great impact on image postprocessing, such as automatic image segmentation. At present, the commonly used offset field correction methods include filtering-based methods, surface fitting-based methods, segmentation-based methods, and histogram-based methods. Among them, the correction method based on the histogram is suitable for offset field correction of different MR images due to its nonparametric characteristics and is widely used in many MR image processing software. A histogram, also known as a mass distribution graph, is a statistical report graph that represents the distribution of data by a series of vertical stripes or line segments of varying heights.

At present, the offset field in MRI is generally considered to be a slowly changing multiplicative field, and the offset field model can be used as follows:

(9) $$\begin{array}{c} B=BA+N\text{.} \end{array}$$

The separation of the offset field *B* and the uncontaminated real image *A* can be achieved by the method of image decomposition.

*p*(*i*) represents the probability that the gray value appears in image *I*, then the entropy of image *I* can be defined by the entropy of the random variable *P* as in the following formula:

(10) $$\begin{array}{c} H\left(I\right)=-\underset{i\in G}{\sum }p\left(i\right)\log\;\left(p\left(i\right)\right)\text{.} \end{array}$$

For a real image without offset field pollution, its entropy value is a fixed value. When it is polluted by the offset field, the probability *p*(*i*) of the image gray value *i* tends to be evenly distributed due to the blurring effect of the offset field, so the entropy of the image polluted by the offset field increases. Therefore, by minimizing the entropy of the image, it can be restored to a real image without offset field contamination.

Entropy generally refers to a measure of the state of certain material systems and the degree to which certain material system states may appear. An entropy-minimizing offset field correction model is introduced into the offset field correction of medical images. In this model, the image degradation process is described by a linear model, which consists of multiplication and an additional component as shown in the following formula:

(11) $$\begin{array}{c} v\left(a\right)=u\left(a\right)m\left(a\right)+b\left(a\right)\text{.} \end{array}$$

*v*(*a*) represents the observed image, *u*(*a*) represents the real image, *m*(*a*) and *b*(*a*) represent the multiplicative and additive components of the offset field. These components are modeled by a combination of smoothly varying basis functions, and the degraded image can be corrected by the inverse of the image degradation model as shown in the following formula:

(12) $$\begin{array}{c} \tilde{u}\left(a\right)=v\left(a\right)m^{-1}\left(a\right)+b^{-1}\left(a\right)\text{.} \end{array}$$

$\tilde{u}\left(a\right)$ is the estimated value of the real image, which can be corrected by minimizing the entropy. The model can maintain the global grayscale statistics while realizing the offset field correction, but the problem of parameter optimization cannot be effectively solved because the degree of freedom of surface search is too large.

In this paper, a model based on LEM offset field correction is used to correct medical images. For the gray value of the *i*th pixel in the image,

(13) $$\begin{array}{c} b_{i}=a_{i}b_{i}+n_{i}\text{.} \end{array}$$

In the formula, *b*_*i*_ represents the gray value of the ith pixel in the observed image, *a*_*i*_ represents the gray value of the ith pixel in the real image, *b*_*i*_ represents the value of the offset field at the ith pixel, and *n*_*i*_ represents the ith pixel. Gaussian noise value for the point. In order to remove the interference of background noise, the model only performs offset field correction for images containing human tissue signals.

### 3.3. Evaluation Criteria for Medical Image Registration

When evaluating the effect of image registration, in addition to directly observing whether the displacement between images is corrected, parameters such as correlation coefficient (CC) and mutual information (MI) can also be used for evaluation. CC reflects the degree of correlation between two images and can be used to evaluate the effect of image registration. The two images are represented by *f*_1_ and *f*_2_. The larger the CC value of the two images, the better the correlation between the two images. CC is defined as follows:

(14) $$\begin{array}{c} CC\left(f_{1},f_{2}\right)=\frac{\underset{a_{i}}{\sum }\left(\left(f_{1}\left(a_{i}\right)-\overset{-}{f_{1}}\right)\left(f_{2}\left(a_{i}\right)-\overset{-}{f_{1}}\right)\right)}{\sqrt{\underset{a_{i}\in \Omega }{\sum }{\left(f_{1}\left(a_{i}\right)-\overset{-}{f_{1}}\right)}^{2}{\left(f_{2}\left(a_{i}\right)-\overset{-}{f_{2}}\right)}^{2}}}\text{.} \end{array}$$

Among them, *f*_1_(*a*_*i*_) represents the gray value of image *f*_1_ at position *a*_*i*_. When used to evaluate the registration effect, the larger the CC value of the two images, the better the registration effect of the two images.

MI represents the statistical correlation between two images and is used in the information field to measure the correlation between two probabilistic variables. Let *H* represent entropy, as in the following equation:

(15) $$\begin{array}{c} MI\left(f_{1},f_{2}\right)=H\left(f_{1}\right)+H\left(f_{2}\right)-H\left(f_{1},f_{2}\right)\text{.} \end{array}$$

Among them, *H*(*f*_1_, *f*_2_) represents the joint entropy of the two images. When used to evaluate the registration effect, the larger the MI between the two images, the higher the registration effect of the image.

For dynamic contrast-enhanced fMRI, the registered images only require that the displacement between images be corrected, while the grayscale changes between images are maintained. And the shape and size of the registered lesion area should remain unchanged for the image containing the tumor. The above-mentioned registration evaluation parameters CC and MI are both calculated according to the corresponding gray values of the images before and after registration. It is suitable for evaluating the registration effect of images with only displacement deformation and no grayscale changes but not for dynamically enhanced fMRI with grayscale changes.

According to the requirements of dynamic-enhanced fMRI registration, the grayscale changes of images before and after registration and the rate of change of lesion area (CRLA) can be used to evaluate the registration effect. The smaller the grayscale change before and after registration, the better the registration effect. CRLA is defined as follows:

(16) $$\begin{array}{c} CRIA=\frac{\left|A_{1}-A_{0}\right|}{\left|A_{0}\right|}\text{.} \end{array}$$

Among them, *A*_0_ represents the size of the lesion area before registration, and *A*_1_ represents the size of the lesion area after image registration. The smaller the CRLA, the smaller the size change of the lesion area after image registration, and the better the registration result.

### 3.4. Breast Dynamic Enhanced fMRI Registration Based on Image Decomposition

Aiming at dynamic enhanced MRI sequences with both grayscale changes and displacement deformations, a nonrigid registration algorithm is proposed in this paper, which must be registered before fMRI can be used to judge benign and malignant breast lesions. However, in the imaging process, if the contrast spreads, the lesion area will produce obvious grayscale changes, and the registration of the dynamic enhanced fMRI of the breast becomes difficult.

With the development of image decomposition technology, the existing image decomposition technology can realize the separation of normal tissue and abnormal tissue in breast dynamic enhanced fMRI. The ROF model based on TV decomposition proposed by scholars can be written as follows:

(17) $$\begin{array}{c} \min{\left\|\forall u\right\|}_{1}+\frac{\mu }{2}{\left\|u-I\right\|}_{2}^{2}\text{.} \end{array}$$

In the formula, *u* represents the structural information of the image, and *I* represents the original image to be decomposed. The model can decompose the image into two parts, one part corresponds to the detailed information in the image, and the other part corresponds to the structural information in the image.

However, when the ROF model is used to decompose the breast dynamic enhanced MRI sequence, the grayscale consistency between the obtained normal tissue image sequences cannot be guaranteed because the model does not impose any constraints on the gray scale between normal tissues. In order to make the gray level between the normal tissue image sequences not change or change very little, that is, the normal image sequences have gray level consistency. This paper introduces constraints on the gray level between normal images. The objective function is as follows:

(18) $$\begin{array}{c} E_{pairwise}=E_{0}+E_{1}+E_{01}\text{.} \end{array}$$

*E*_0_ represents two dynamic enhanced MRIs of the breast; *E*_1_ and *E*_2_ represent abnormal tissue images in dynamic enhanced MRI of the breast.

In order to separate the normal tissue and abnormal tissue in the breast dynamic enhanced MRI, the gray histogram of the breast region in the normal tissue image obtained by decomposing should be similar to the first large peak of the gray histogram in (a), as shown in Figure 5

As shown in Figure 5, the displacement deformation between medical images will bring trouble to the subsequent analysis and processing of the images, so registration needs to be performed before further processing. Grayscale refers to the use of black tones to represent objects, that is, to use black as the base color and to display images with different saturations of black. Commonly used nonrigid registration algorithms for medical images include nonrigid registration algorithms based on optical flow field and nonrigid registration algorithms based on FFD. However, for dynamic contrast-enhanced MRI with grayscale changes, direct registration using these methods will lead to distortion of the registered image, especially the tumor area will be severely distorted, which will greatly affect the subsequent analysis.

## 4. Nursing Experiment of Breast Cancer Patients with Lymphomegaly Based on fMRI

### 4.1. Investigation of Breast Cancer Patients with Lymphomegaly

In this paper, 60 patients admitted to the lymphatic surgery ward of a hospital from December 2018 to January 2019 were selected as the research subjects, and the researchers initially screened and included the admitted patients according to the inclusion and exclusion criteria. 60 people were divided into the control group and intervention group. The control group was group *A*, and the intervention group was group *B*. The 60 patients were all based on the treatment that had relapsed problems.

The control group was given routine nursing measures, and the intervention group was given the fMRI program on the basis of routine nursing. The original data were entered and analyzed using SPSS16.0 statistical software. The patients are all female, and the basic information about the patients is shown in Table 1.

As shown in Table 1, the patients in this experiment are all female, of which 13 and 15 were aged 45 to 50 in Group *A* and Group *B*, and 17 and 15 were aged 50 to 55, respectively. It can be seen that there is little difference in age between the two groups.

In terms of the course of the lymphatic disease, the number of patients with lymphedema was 2 years to 4 years, 14 and 17 people, respectively, and 16 and 13 people were 4 years to 6 years. The difference is not much. This shows that the difference between the experimental data in this paper is very small, which can ensure the real reliability of the experiment.

In this paper, in order to understand which measures the patients took care of before the experiment, the two groups were investigated and analyzed, as shown in Figure 6.

As shown in Figure 6, after the occurrence of edema, the patients usually receive care and intervention through simple massage, exercise therapy, western medicine treatment, and traditional Chinese medicine treatment. Among them, 10 people in group *A* were treated by simple massage, and 6 people in group *B*. There are 6 people in group *A* and 5 people in group *B* through exercise therapy; 9 people in group *A* and 12 people in group *B* through western medicine treatment; 5 people in group *A* and 7 people in group *B* through traditional Chinese medicine treatment. Because they think it will save their time and not affect their work. But the effect of treatment is not very good, the treatment effect of the four methods is less than 50%, so the quality of nursing is not high.

### 4.2. Contrast Experiment Before and After the Two Groups of Experiments

Effective care of patients with breast cancer-related lymphedema after surgery can improve the number and severity of lymphedema-related symptoms. After 6 months of nursing, the patients were investigated and analyzed again to understand their nursing quality and the severity of edema in the two groups before and after the experiment was investigated, as shown in Figure 7:

As shown in Figure 7, before the experiment, there were 10 people with very serious edema in group *A*, accounting for 33.3%, and 10 people with more serious edema, accounting for 33.3%, 5 people are generally serious, accounting for 16.7%, and 5 people are not serious; the percentage is 16.7%. In group *B*, 12 people had very serious edema, accounting for 40%, 11 people had more serious edema, accounting for 36.6%, 4 people generally had severe edema, accounting for 13.3%, and 3 people were not serious; the percentage was 10.1%. It can be seen that the number of patients with severe edema in the two groups before the experiment is still more, and the difference between the two groups is not obvious.

After the experiment, there were 9 people with very serious edema in group *A*, 8 people with more serious edema, 7 people with general serious edema, and 6 people with less serious edema. After the experiment in group *B*, the number of serious and very serious cases was 4, the more serious was 3, the general serious was 3, and the nonsevere was 20, indicating that the nursing program of group *B* played a great role.

### 4.3. Experiments in Breast Image Lesion Recognition Based on FMRI Technology

The breast dynamic contrast-enhanced fMRI used in this experiment was obtained from the imaging data of the two groups of patients. The acquisition equipment is the 1.5 T and 3.0 T magnetic resonance superconductors of General Company, and the acquisition and scanning methods are transverse and sagittal scanning. In order to ensure the reliability of the results, the experiment used ultrasound, X-ray, and fMRI to reexamine six patients with the same postoperative time and all of the lesions recurred. The results are shown in Tables 2–4.

As shown in Tables 2–4, usually, ultrasound and X-ray examinations are not very accurate in distinguishing scar tissue and tumor recurrence in patients with breast cancer lymphedema after treatment. Soft tissue resolution, multidirectional multiparameter imaging, and minimal radiation damage are all advantages of breast fMRI imaging. After treatment, fMRI can effectively detect postoperative tumor recurrence and postoperative scar tissue, and fMRI can detect residual or postoperative recurrent tumor lesions with a sensitivity of more than 90%.

The process of image acquisition is that after the patient is lying down in the prone position, the first scan is performed to obtain the image, and then the contrast agent is injected, and then the enhanced scan image is started, and the temporal resolution of the enhanced scan is about 60 s. In the experiment, this paper only analyzes and processes the lesion area, and the size of the lesion area is extracted according to the size of the breast lymph, as shown in Figure 8.

As shown in Figure 8, in this study, the TV decomposition model was used to deconstruct dynamic enhanced breast MRI into normal and pathological tissue images. The displacement deformation field between the images is extracted by registration, and the original breast dynamic enhanced fMRI is registered with the deformation field so as to achieve accurate breast dynamic enhanced fMRI registration.

The changes between breast dynamic enhanced fMRI reflect the diffusion information of contrast agents in breast tissue over time, which can assist in the differentiation of benign and malignant lesions. Therefore, it is very important to maintain the grayscale consistency of the corresponding phase images before and after registration, as shown in Figure 9.

As shown in Figure 9, the shape of the lesion area is one of the important information for distinguishing benign and malignant lesions, so the preservation of the lesion area after registration is very important. Compared with the original image, the shape of the lesion area in the registered breast dynamic contrast-enhanced fMRI is almost not distorted, which indicates that the registered breast dynamic contrast-enhanced fMRI can well maintain the shape of the lesion. From the experimental results, it can be seen that the size of the registered lesion area has little change compared with the original image, which shows that the registered lesion area has changed little, but the change is small.

Using the registration method proposed in this paper to register the dynamic contrast-enhanced fMRI of the breast enables the displacement between images to be corrected. It can ensure that the lesion area in dynamically enhanced fMRI of the breast after registration will not be distorted, and at the same time, it can maintain the same gray level change information between the registered image and the original image.

## 5. Conclusions

With the increasing success rate of breast cancer surgery in recent years, people are no longer satisfied with the improvement of survival but pay more attention to the quality of life after treatment. Lymphedema occurs in many patients. Although it does not seem to be a serious disease, it has caused great trouble to the patients' lives. Therefore, it is necessary to study the nursing care of patients with edema after treatment. With the development of fMRI technology, the identification rate and localization accuracy of lesions are also getting higher and higher. Therefore, this paper is mainly based on fMRI technology to study the nursing care of patients with breast cancer lymphedema after treatment. The application of fMRI technology will improve the effect of nursing care for patients after treatment. In order to more accurately identify the lesions, this paper proposes an image registration method in the method part, which can improve the functional effect of fMRI technology in identifying images. In order to verify that fMRI technology can assist the nursing care of patients after treatment, this paper conducted experiments on two groups of patients with different nursing methods in the experimental part. The results showed that the nursing effect of the patients in the fMRI technology group was better than that of the control group. The image processing based on image registration method has a higher registration rate so as to accurately find the lesion area and prevent a recurrence. In this paper, only 60 patients were investigated in the experiment, which made the data of the experiment scientific. Therefore, in future work, more patients should be compared and the conclusions drawn would be more rigorous.

## Figures and Tables

**Figure 1:** Traditional care for lymphedema in breast cancer.

**Figure 2:** Advantages of fMRI technology.

**Figure 3:** Image registration.

**Figure 4:** Overall schematic of SPM processing fMRI data.

**Figure 5:** Grayscale histograms of the mammary gland region in the original and decomposed normal tissue. (a) Grayscale histogram of the original image. (b) Grayscale histogram of the decomposed image.

**Figure 6:** Traditional nursing measures and efficacy. (a) Traditional nursing measures. (b) Effectiveness of traditional nursing measures.

**Figure 7:** Severity of edema in the two groups (a) before the experiment and (b) after the experiment.

**Figure 8:** Quantification results of grayscale consistency of raw image sequences and normal tissue image sequences.

**Figure 9:** The rate of change of the lesion area in the images before and after the algorithm in this paper is registered. (a) The rate of change of the lesion area of the image before registration. (b) The rate of change of the lesion area of the image after registration.

**Table 1:** Basic information of patients.

Project	Overall	Group *A*	Group *B*
Age	45–50	13	15
	50–55	17	15
Course of disease (years)	2–4	14	17
	4–6	16	13
Edema site	Left	12	16
	Right	18	14
Predisposing factors	Have	10	9
	None	20	21

**Table 2:** Accuracy and sensitivity of ultrasound in identifying recurrent lesions.

Patients	Postoperative time (months)	Accuracy (%)	Sensitivity (%)
Patient 1	3–6	56	51
Patient 2	3–6	54	62
Patient 3	3–6	55	61
Patient 4	3–6	53	58
Patient 5	3–6	52	57
Patient 6	3–6	49	53

**Table 3:** Accuracy and sensitivity of X-ray in identifying recurrent lesions.

Patients	Postoperative time (months)	Accuracy (%)	Sensitivity (%)
Patient 1	3–6	62	58
Patient 2	3–6	67	66
Patient 3	3–6	66	63
Patient 4	3–6	63	57
Patient 5	3–6	64	59
Patient 6	3–6	65	62

**Table 4:** Accuracy and sensitivity of fMRI for discriminating recurrent lesions.

Patients	Postoperative time (months)	Accuracy (%)	Sensitivity (%)
Patient 1	3–6	87	92
Patient 2	3–6	89	90
Patient 3	3–6	92	95
Patient 4	3–6	88	96
Patient 5	3–6	93	94
Patient 6	3–6	91	91

## Data Availability

The datasets generated during and/or analyzed during the current study are not publicly available due to sensitivity and data use agreement.

## References

[1] Ziv E., Cauley J., Morin P. A. (2017). Saiz R, Browner WS. Association between the T29⟶C polymorphism in the transforming growth factor *β*1 gene and breast cancer among elderly white women: the study of osteoporotic fractures. *Journal of the American Medical Association*.

[2] Lautrup M. D., Thorup S. S., Jensen V. (2017). Male breast cancer: a nation-wide population-based comparison with female breast cancer. *Acta Oncologica*.

[3] Retsky M., Bonadonna G., Demicheli R., Folkman J. (2017). Hypothesis: induced angiogenesis after surgery in premenopausal node-positive breast cancer patients is a major underlying reason why adjuvant chemotherapy works particularly well for those patients. *Breast Cancer Research*.

[4] Yuka A., Shinichiro K., Wataru G., Sayaka T., Tamami M., Tsutomu T. (2017). Expression and clinical significance of androgen receptor in triple negative breast cancer. *Cancers*.

[5] Harris E., Small W. (2017). Intraoperative radiation therapy for breast cancer. *Surgical Oncology Clinics of North America*.

[6] Alexis H. A., Barbara M. M., Michel C. M. (2017). fMRI of simultaneous interpretation reveals the neural basis of extreme language control. *Cerebral Cortex*.

[7] Liu T. T., Nalci A., Falahpour M. (2017). The global signal in fMRI: nuisance or Information?. *NeuroImage*.

[8] Ali K., Ata E., Abbas B. F. (2017). Classification of patients with MCI and AD from healthy controls using directed graph measures of resting-state fMRI. *Behavioural Brain Research*.

[9] Chen X., Lu B., Yan C. G. (2017). Reproducibility of R-fMRI metrics on the impact of different strategies for multiple comparison correction and sample sizes. *Human Brain Mapping*.

[10] Szaflarski J. P., Gloss D., Binder J. R. (2017). Practice guideline summary: use of fMRI in the presurgical evaluation of patients with epilepsy. *Neurology*.

[11] Tixier H., Bermudez F., Iyer D. (2018). Impact of image preprocessing methods on the robustness of MRI-based radiomic classifiers for glioblastoma. *Medical Physics*.

[12] Prem J. T., Sukanya P., Madhavi T. (2020). Brain tumor discovery using image preprocessing. *International Journal of Research in Pharmacy and Science*.

[13] Ma H., Wang K. (2019). A hybrid method for underwater image preprocessing. *International Journal of Sciences*.

[14] Bindu G. H., Reddy P., Murty M. R. (2018). Image preprocessing of abdominal CT scan to improve visibility of any lesions in kidneys. *Journal of Theoretical and Applied Information Technology*.

[15] Liu K., Bi Y., Wang M. (2018). Cotton image preprocessing based on combination of edge detection and noise classification. *IPPTA: Quarterly Journal of Indian Pulp and Paper Technical - A*.

[16] Puspaningrum E. Y., Alit R. (2018). Surjohadi. Image preprocessing with symmetrical face images in face recognition and regression classification. *International Journal of GEOMATE*.

[17] Patel I., Patel S., Patel A. (2018). Analysis of various image preprocessing techniques for denoising of flower images. *INTERNATIONAL JOURNAL OF COMPUTER SCIENCES AND ENGINEERING*.

[18] Susan E. (2017). Chemotherapy-induced amenorrhea and fertility in women undergoing adjuvant treatment for breast cancer. *Cancer Control*.

[19] Wei L., Liu T. T., Wang H. H. (2011). Hsp27 participates in the maintenance of breast cancer stem cells through regulation of epithelial-mesenchymal transition and nuclear factor-*κ*B. *Breast Cancer Research*.

[20] Brunelle C. L., Swaroop M. N., Skolny M. N., Asdourian M. S., Sayegh H. E., Taghian A. G. (2018). Hand edema in patients at risk of breast cancer–related lymphedema: health professionals should take notice. *Physical Therapy*.

